# Determination of Scopolamine Distribution in Plasma and Brain by LC-MS/MS in Rats

**DOI:** 10.1155/2022/8536235

**Published:** 2022-09-30

**Authors:** Juan Chen, Anjing Lu, Daopeng Tan, Qianru Zhang, Yanliu Lu, Lin Qin, Yuqi He

**Affiliations:** ^1^Guizhou Engineering Research Center of Industrial Key-technology for Dendrobium Nobile, Zunyi Medical University, Zunyi, Guizhou 563000, China; ^2^Joint International Research Laboratory of Ethnomedicine of Ministry of Education, Zunyi Medical University, Zunyi, Guizhou 563000, China

## Abstract

Scopolamine, as a tropane alkaloid found in plants such as belladonna and datura, is used clinically as a transdermal patch and is highly neurotoxic. This study aimed to develop a simple, sensitive, and selective LC-MS/MS method for the determination of the content and distribution of scopolamine in rat plasma and brain after drug administration. In our study, sample pretreatment consisted of protein precipitation with acetonitrile followed by nitrogen blow concentration. Gradient elution of scopolamine and internal standard was performed on a ZORBAX Eclipse Plus C18 (2.1*∗*100 mm, 3.5 *μ*m) column with water containing 0.1% formic acid (*v/v*) and acetonitrile as a mobile phase. Those samples were quantified in ESI positive ion mode using an API 4000 triple quadrupole mass spectrometer. The results showed that scopolamine was linear in the calibration range of 2–2500 ng/mL, and the selectivity, accuracy, precision, matrix effect, stability, and recovery of the method were within acceptable limits. The method has been validated and has been successfully used for toxicokinetic studies of scopolamine. After intraperitoneal injection, the time to peak toxic concentrations of scopolamine in rats was 0.5 h. The concentrations of scopolamine in the hippocampus and cortex were much higher than those in the striatum, indicating that the likely targets of its neurotoxic damage were the hippocampus and cortex. Overall, this study provides the basis for the neurotoxicity of scopolamine and provides a reference for its toxicokinetic studies.

## 1. Introduction

Scopolamine is an alkaloid found mainly in belladonna and datura [1]. Currently, scopolamine is mainly used as a competitive inhibitor of nonselective muscarinic acetylcholine receptors with potent peripheral antimuscarinic properties and central sedative and antiemetic effects [2]. In the clinic, the routes of administration of scopolamine include transdermal patches, oral administration, and injection, but the bioavailability of patches and oral administration is limited. Its absolute bioavailability for oral administration has been reported to range from 3% to 27% [3]. So far, scopolamine has been widely used in anesthesia, analgesia, antimotion sickness, antiepileptic drug detoxification [4], antiparkinsonism [5], and postoperative prevention of nausea and vomiting [6].

Scopolamine has relatively powerful pharmacological effects, but it has also been implicated in toxicology-related studies. Because of its high lipid solubility, it is highly susceptible to neurological toxicity by crossing the blood-brain barrier [7]. Whether used clinically as a transdermal patch or functioning as the main component in the plant, scopolamine has certain toxic side effects. Its toxic symptoms are mainly neurotoxic, mostly due to misuse, intentional or unintentional abuse (victim control, dilution of illicit drugs), accidental ingestion of parts of the plant (mainly in children), and its presence in contaminated food [8, 9]. A 66-year-old female patient was reported to have developed anticholinergic toxicity including delayed awakening, loss of consciousness, unresponsiveness, acute manic episodes, paranoia, dilated pupils, and tachycardia after a preoperative transdermal patch of scopolamine was applied behind the ear to prevent postoperative gastrointestinal adverse effects [10]. Scopolamine is an alkaloid that threatens life and health, so its quantification is of great importance in pharmacology and toxicology.

At present, many methods have been developed to quantify scopolamine, including high performance thin-layer chromatography (HPTLC) [11], gas chromatography-mass spectrometry (GC-MS) [12], high performance liquid chromatography (HPLC) [13], capillary electrophoresis [14], high performance liquid chromatography-tandem mass spectrometry (LC-MS/MS) [8, 15], and radioimmunoassay [16]. Among these reported quantitative analysis methods, LC-MS/MS is the most commonly used. The principle of LC-MS/MS is that the sample is first carried by the mobile phase in the liquid phase module into the column for separation, and the separated compound enters the mass spectrum, where it is ionized in the ion source, and then scanned by the primary mass spectrum into the collision cell, where the molecular ions are collisionally cleaved to form product ions into the second mass spectrum, and finally into the detector for detection [17, 18]. Compared with other detection methods, LC-MS/MS has the advantages of high sensitivity, high selectivity, and high efficiency and requires less biological matrix, which is suitable for the simultaneous determination of multicomponent compounds, and its application in both pharmacokinetic and toxicological studies is becoming more and more dominant [19].

So far, most of the methods developed for the analysis of scopolamine have been used to quantify the scopolamine content in plants, foods, and humans, but research data on the quantitative detection of scopolamine in biological samples are limited. In addition, although scopolamine has been used in clinical applications for many years, it is an alkaloid that threatens human health and life, and there are few reports and studies on its toxicity at home and abroad. Therefore, this study aimed to develop a simple, sensitive, and selective LC-MS/MS method for the determination of scopolamine content and distribution in rat plasma and brain tissue. This method has been successfully applied to determine the content of intense neurotoxicity in rats following a single intraperitoneal injection of a large dose of scopolamine.

## 2. Materials and Methods

### 2.1. Chemicals and Reagents

Scopolamine hydrobromide (purity >98%) was purchased from Chengdu Alfa Biotechnology Co. Ltd. (Chengdu, China) and reference standard (purity >98%) was purchased from the Henan standard material R&D Center Co. Ltd. (Henan, China). Pseudoephedrine hydrochloride (internal standard) (purity >98%) was purchased from the National Institute for Food and Drug Control (Beijing, China). Acetonitrile, methanol, and formic acid (LC/MS grade) were purchased from Thermo Fisher Scientific Co. Ltd. (Shanghai, China). All the other reagents were of analytical grade.

### 2.2. LC-MS/MS Quantitative Analysis Conditions

#### 2.2.1. Instrument and Equipment

Liquid chromatography API 4000™ triple quadrupole tandem mass spectrometer (AB SCIEX, USA) was used for chromatographic separation and quantitative determination.

#### 2.2.2. Chromatographic Conditions

The chromatographic elution was performed on an Agilent ZORBAX Eclipse Plus C18 column (2.1*∗*100 mm, 3.5 *μ*m) with a column temperature of 25°C. Mobile phase A was a 0.1% formic acid solution, and mobile phase B was acetonitrile. The elution gradient was 0–2 min, 90% A; 2-3 min, 90% A⟶50% A; 3–6 min, 50% A; 6-7 min, 50% A⟶90% A; 7–10 min, 90% A at a flow rate of 0.3 mL/min. The injection volume was 2 *μ*L.

#### 2.2.3. Mass Spectrometry Conditions

The scopolamine hydrobromide reference solution and internal standard solution were configured to a final concentration of 500 ng/mL by adding 100 *μ*g/mL to water-methanol (50 : 50, *v/v*), respectively. The initial mass spectrometric conditions for scopolamine and the internal standard were obtained by injection into LC-MS/MS and used for method development.

The mass spectra were performed using an electrospray ionization source (ESI) with a positive ion multiple reaction detection mode (MRM). The ESI-MS/MS operating parameters used in the method were set as follows: ion spray voltage of 5500 V, curtain gas 25 psi, ion source gas1 40 psi, ion source gas2 45 psi, temperature 450°C, and collision gas 8. Other parameters are adjusted for individual chemical substances.  Table 1 shows the information on the precursor and product ions of scopolamine with internal standards.

### 2.3. Preparation of Solutions

A certain mass of scopolamine hydrobromide control and internal standard were weighed and dissolved in methanol (concentration of 1 mg/mL and 100 *μ*g/mL, respectively) as the initial solution, and then the initial solution of scopolamine was diluted to 100 *μ*g/mL and 2 *μ*g/mL with 50% methanol as the stock solution, respectively. Subsequently, the scopolamine control solution was diluted with 50% methanol to 9 concentrations of 60 ng/mL, 150 ng/mL, 300 ng/mL, 1500 ng/mL, 7500 ng/mL, 15000 ng/mL, 30000 ng/mL, 60000 ng/mL, and 75000 ng/mL as calibration solutions for the calibration curve. In addition, an appropriate amount of the initial solution of the internal standard in 50% methanol was used to prepare the internal standard working solution with a final concentration of 1 *μ*g/mL.

Scopolamine stock solution was taken and diluted with 50% methanol into 4 concentrations of 60 ng/mL, 150 ng/mL, 7500 ng/mL, and 56250 ng/mL as the quality control (QC) working solutions. All the above solutions were prepared and stored at 4°C for backup.

### 2.4. Preparation of Plasma and Brain Samples

#### 2.4.1. Plasma Samples

To 50 *μ*L of rat plasma, 10 *μ*L of internal standard working solution and 240 *μ*L of acetonitrile were added. Then, the samples were vortexed and mixed for 60 s and centrifuged at 16000 rpm for 5 min at 4°C. 20 *μ*L of supernatant was placed in a new centrifuge tube. The supernatant was evaporated to dryness using nitrogen at room temperature, redissolved by adding 50% acetonitrile (1 : 1, *v/v*) 200 *μ*L, sonicated, and vortexed for 60 s, and then centrifuged at 16000 rpm for 10 min at 4°C. Finally, 50 *μ*L of the supernatant was injected into LC-MS/MS for analysis.

#### 2.4.2. Brain Homogenate Samples

Samples of each brain region (hippocampus, striatum, cortex) were removed, placed in liquid nitrogen, weighed, and recorded. Prechilled saline was added to the tissue in the ratio of 1 g : 6 mL, and then 2 small magnetic beads were added and homogenized at 50 HZ for 2 min at 4°C until no particles were visible to the naked eye. After centrifugation at 4500 rpm for 10 min at 4°C, the supernatant was taken to obtain the brain homogenate sample, which was stored at −80°C.

The brain homogenate samples obtained above were processed according to the method under 2.4.1 “Plasma sample.”

### 2.5. Validation of Analytical Methods

#### 2.5.1. Selectivity

Six blank plasma and brain homogenates from different sources were processed and sampled according to the method under item 2.4 and analyzed by the LC-MS/MS method under item 2.2. The method was examined to see if it could distinguish scopolamine and internal standard from endogenous components of the biological matrix or other components of the drug.

#### 2.5.2. Calibration and Lower Limit of Quantification

The calibration curve model was determined by linear regression using weighted least squares with the concentration of scopolamine as the horizontal coordinate and the ratio of the peak area of scopolamine to the peak area of the internal standard as the vertical coordinate.

The signal-to-noise ratio (S/N) of >10 for the lower limit of quantification and S/N > 3 for the limit of detection were required. The linear method of the calibration curve was used to estimate the concentration of the unknown sample. A total of three calibration curves were evaluated in this methodological validation.

#### 2.5.3. Accuracy and Precision

Four concentrations: 60 ng/mL, 150 ng/mL, 7500 ng/mL, and 56250 ng/mL, were used to examine the precision and accuracy of the method. The intraday accuracy and precision of the method were assessed by analyzing blank plasma and brain homogenate samples at each calibration curve level. Interday accuracy and precision validation were assessed separately over three days. The quality control sample concentrations were determined from the accompanying standard curves, and the final ratio of the mean of the measured concentrations to the labeled concentrations was used to express the relative error (RE) for accuracy. The ratio of the standard deviation of the measured concentration to the mean value of the measured concentration is the relative standard deviation (RSD), which is used to express precision.

#### 2.5.4. Matrix Effect and Recovery

Six blanks of different sources of plasma and brain tissue homogenates were added to 240 *μ*L of acetonitrile, vortexed, and mixed for 60 s. After centrifugation, 200 *μ*L of the supernatant was injected into a new centrifuge tube and blown dry under nitrogen. The sample was analyzed by adding 10 *μ*L of low and 10 *μ*L of high-quality control solution, 10 *μ*L of internal standard solution, 180 *μ*L of 50% acetonitrile, vortexing, sonication for 60 s, and centrifugation at 16000 rpm for 10 min at 4°C. 50 *μ*L of the supernatant was used for sample analysis, and the peak areas of the matrix samples were A_Scop_ and A_IS_, respectively. 180 *μ*L of the compound solution was also used for sample analysis. The matrix effect of analytes was calculated by the ratio of scopolamine to internal standard peak area in matrix samples and the ratio of scopolamine to internal standard peak area in pure solution samples (A_Scop_/A_IS_)/(C_Scop_/C_IS_).

High- and low-concentration QC samples were prepared and analyzed according to the method below item 2.4.1. The peak area ratio B_Scop_/A_Scop_ (or B_IS_/A_IS_) of scopolamine (or internal standard) of the control sample to that of the matrix sample is the recovery of scopolamine (or internal standard).

#### 2.5.5. Stability

Stability was investigated using QC samples of low and high concentrations. Refrigeration stability, repeated freeze-thaw stability, and autosampler stability were evaluated to demonstrate the reliability and usefulness of the method in the study. Refrigeration stability was determined by adding the quality control working solution to plasma and brain homogenate, respectively, at 4°C for 24 h and 48 h, then feeding the samples for analysis according to the sample processing method in item 2.4. For repeated freeze-thaw stability, the main purpose was to examine whether the stability of biological samples changed after primary and secondary freeze-thaw. For autosampler stability, the treated samples were placed in an autosampler with a set temperature of 15°C and analyzed after 12 h, and then the relative standard deviation was calculated.

### 2.6. Pharmacokinetic Study

#### 2.6.1. Experimental Animals

10 Sprague–Dawley (SD) rats (male, 200–250 g) were purchased from Hunan Slike Jingda Experimental Animal Co. Ltd (Hunan, China; Certificate No. SCXK2019-0004). All rats were housed at a temperature of 23°C and a 12 h/12 h light/dark cycle. Rats were fed and watered freely, but fasted the night before the start of the experiment. All rats were acclimatized and fed for 3 days before the start of the experiment.

#### 2.6.2. Sample Collection

Scopolamine dissolved in saline was given intraperitoneally to 10 rats at a single dose of 400 mg/kg (this dose was derived from our previous study on the acute toxicity of scopolamine, which is not yet published), and orbital blood sampling was performed at 0 h, 0.083 h, 0.167 h, 0.25 h, 0.5 h, 0.75 h, 1 h, 1.5 h, and 2 h after administration. Blood samples from all rats were collected in 1.5 mL centrifuge tubes (containing 1% sodium heparin) and then immediately centrifuged at 4500 rpm for 15 min at 4°C. The supernatant was removed to obtain plasma, which was stored at −80°C.

The brain tissues (hippocampus, striatum, cortex) of rats were isolated after blood sampling at 2 h, washed with prechilled saline until no blood color was observed, and blotted dry with filter paper. After precise weighing, the brain tissue samples were homogenized according to 2.4.2.

## 3. Results and Discussion

### 3.1. Optimization of Chromatographic and Mass Spectrometric Parameters

ESI has high polarity and was therefore chosen for the ionization of scopolamine and internal standards in this study [15]. To obtain a higher relative abundance of precursor and product ions, the cone voltage and collision energy were optimized in this study. The highest abundance and the content of the protonated molecule [*M* + *H*]^+^ were detected in full scan mode at *m*/*z* 304.2 for scopolamine and *m*/*z* 166.3 for the internal standard. In the product ion scan, the high abundance fragment ions of 138.1, 156.1, and 120.9 for scopolamine and 148.1 for the internal standard, respectively, were finally selected as the highest abundance fragment ions for subsequent quantitative analysis of scopolamine and the internal standard. In addition, the capillary temperature, ion spray voltage, and nebulizer of the mass spectrometry were optimized to obtain the best results. The specific results are shown in Table 1.

For the liquid phase, different chromatographic conditions were investigated to optimize peak shape, retention time, and sensitivity of detection for both the column and mobile phase. First, we chose an Agilent Zorbax Eclipse Plus C18 column, which can withstand a higher percentage of the aqueous phase and better retain alkaline compounds [20]. Various compositions of mobile phases, including water-methanol and water-acetonitrile, as well as different proportions of formic acid or ammonium acetate, were tested to achieve good peak shapes and ionization [20–22]. The addition of an appropriate amount of formic acid and ammonium acetate to the mobile phase can make the alkaloids exist in the form of ions, which can reduce the distortion and splitting of peaks caused by the coexistence of ionic forms and molecular forms of compounds and also prevent the trailing of peaks. However, excess buffer salts or excess ionization in the solution can contaminate the column as well as the mass spectrometer [15]. Therefore, 0.1% formic acid water-acetonitrile was finally chosen as the mobile phase in this study to obtain a better peak shape and sensitivity.

### 3.2. Validation of LC-MS/MS Methods

#### 3.2.1. Selectivity

The method is highly selective, and the results are shown in Figure 1. The responses of endogenous interference peaks in blank plasma and blank brain tissue were less than 5% for the corresponding retention times of scopolamine and internal standard. Under the assay conditions, endogenous substances from plasma and brain tissue did not interfere with the sample determination. The experimental results showed that scopolamine and the internal standard could be well distinguished, indicating that the method has good specificity.

#### 3.2.2. Calibration Curve and Lower Limit of Quantification

The effective concentrations of scopolamine in rat plasma and brain tissue ranged from 2 to 2500 ng/mL, and the calibration curve was linear in this range.  Table 2 details the regression equations for the calibration curves and the correlation coefficients associated with scopolamine. Three calibration curves were prepared in parallel, and the concentrations of the three standard curves corrected for back-calculation of the standard samples were within 15% of the indicated values, the lower limit of quantification was within 20%, and the linear correlation coefficients (*r*) of the standard curves for plasma and brain tissue samples were all greater than 0.992. The results show that scopolamine has good linearity in the calibration range and that the standard curve can accurately quantify the concentration of scopolamine in plasma and brain tissue.

#### 3.2.3. Accuracy and Precision

The intraday and interday accuracy and precision results of scopolamine in rat plasma and brain tissue at the four QC concentration levels are shown in Table 3. According to the requirements, the accuracy of all QC samples was within ±15% of the indicated values, the accuracy of the lower limit of quantification was within ±20% of the indicated values, the precision was less than 15%, and the precision of the lower limit of quantification was less than 20%.

The results met the requirements. It showed that the method was reproducible and the determined results were accurate and reliable.

#### 3.2.4. Matrix Effect and Recovery

The results of the matrix effect and recovery of scopolamine in plasma and brain tissue samples are shown in Table 4. The mean recovery of scopolamine in both plasma and brain tissue samples exceeded 92.87% at both low- and high-quality control concentrations, and the RSDs were less than 15%. In addition, the mean values of the matrix effect of low- and high-quality control samples of scopolamine in plasma samples and brain tissue samples ranged from 87.13% to 114.01%, with RSD within 11.40%. This indicates that the assay is not affected by ion enhancement or inhibition in rat plasma and brain tissue samples, and there is no significant matrix effect.

#### 3.2.5. Stability

The short-term refrigeration (Table 5), repeated freeze-thaw stability, and autosampler stability (Table 6) of the low and high concentrations QC solutions were examined. As shown in the results, after short-term freezing, the accuracy of scopolamine in both high- and low-concentration QC samples was above 91.25%, and the RSD was within 15% for both. After freeze-thawing once, the accuracy of scopolamine in low-and high-concentration QC samples was in the range of 91.09% to 115.70% with RSD less than 9.44%. However, after repeated freeze-thawing twice, the accuracy of the low QC concentration of plasma samples did not meet the requirement, and the accuracy of QC samples at this concentration was much greater than ±15% of the indicated value.

Therefore, to ensure the accuracy of the measurement results, repeated freeze-thawing should be avoided for plasma samples a second time. For brain homogenate samples, after repeated freeze-thawing twice, the accuracy of low and high-concentration quality control samples ranged from 106.54% to 86.23%, with a precision of less than 6.35%. The accuracy of scopolamine in the samples was within ±15% of the labeled value after 12 h of placement in the autosampler, and the RSD was all less than 11.71%.

The results showed that the samples had good stability after short-term refrigeration, freeze-thawing once, and 12 h in the autosampler under the above conditions, ensuring that stability-related problems would not interfere with the determination of scopolamine concentrations in plasma and brain tissue. However, repeated freeze-thawing of the samples, especially twice, should be avoided during the experiment.

### 3.3. Pharmacokinetic Study

To verify the usability of the method, the study first examined plasma (Figure 2) and brain tissue (Figure 3) drug concentrations in rats after intraperitoneal injection of scopolamine to better elucidate the blood concentration of scopolamine at toxic doses of administration and its distribution in the brain.

Firstly, the LC-MS/MS method established and validated above was used to determine the plasma drug concentration versus time in rats at 0 h, 0.083 h, 0.167 h, 0.25 h, 0.5 h, 0.75 h, 1 h, 1.5 h, and 2 h of intraperitoneal injection of larger doses of scopolamine, and the results are shown in Figure 2. Among the 10 rats, 3 rats reached the peak at 0.25 h after administration (Figure 2(b)), 5 rats reached the peak at 0.5 h after administration (Figure 2(c)), and 2 rats reached the peak at 0.75 h after administration (Figure 2(d)), but scopolamine was gradually metabolized in all rats after 1 h of administration. The results showed that the blood concentration of scopolamine in rats showed individual variability, and the peak time of scopolamine blood concentration after intraperitoneal injection ranged from 0.25 h to 0.75 h, but mainly reached the peak at 0.5 h.

Similarly, the concentration of scopolamine in the brain after 2 h of intraperitoneal injection was determined by LC-MS/MS, and the results are shown in Figure 3(a). Because of the higher dose administered, the concentration of scopolamine in vivo was also relatively high. The concentrations of scopolamine in rat hippocampus, striatum, and cortex tissues were 3.54 × 10^5^∼1.05 × 10^6^ ng/g, 4.31 × 10^5^∼1.80 × 10^6^ ng/g, 3.31 × 10^5^∼3.01 × 10^6^ ng/g, respectively. The differences between the lowest and highest concentrations were about 3, 4, and 9 times, respectively, which suggested that there is also some individual variability in the exposure of scopolamine in rat brains. Next, the drug concentrations in the hippocampus, striatum, and cortex of rats after a single intraperitoneal injection of scopolamine for 2 h were correlated with plasma drug concentrations, and the results are shown in Figures 3(b)–3(d). Scopolamine concentrations in hippocampus and cortex tissues showed a significant positive correlation with plasma drug concentrations, with the most significant correlation in the hippocampus (*P*-value 0.00023), while the striatum did not correlate strongly with plasma drug concentrations. It indicates that the concentrations of scopolamine in the hippocampus and cortex tissues are much higher than those in the striatum, and its neurotoxic damage sites may be the hippocampus and striatum, which is consistent with the previous findings [1, 23, 24]. This result also suggests that the exposure to scopolamine in brain tissue may correlate with the concentration of scopolamine in plasma and that the concentration of scopolamine in plasma may determine its concentration in the brain. However, further studies are needed to confirm this.

## 4. Conclusion

In this study, a simple, rapid, accurate, and sensitive LC-MS/MS method was developed and validated for the toxicokinetic analysis of scopolamine, mainly in rat plasma and brain tissue. The results showed that the peak toxic concentration of scopolamine in rats was mainly 0.5 h after intraperitoneal injection and was gradually metabolized after 1 h. The concentration of scopolamine is much higher in the hippocampus and cortex tissues than in the striatum. Therefore, the site of injury for scopolamine neurotoxicity may be the hippocampus and striatum, and the concentration in plasma may determine its concentration in the brain.

## Figures and Tables

**Figure 1:** MRM chromatograms of blank plasma (a), plasma sample containing internal standard (1) and scopolamine (2) (b), blank brain (c), and brain tissue sample containing internal standard (1) and scopolamine (2) (d).

**Figure 2:** Blood concentration-time curves of 10 rats after a single intraperitoneal injection of scopolamine for 2 h (a), with peak times of 0.25 h in 3 rats (b), 0.5 h in 5 rats (c), and 0.75 h in 2 rats (d).

**Figure 3:** The concentration of scopolamine in the hippocampus, striatum, and cortex at 2 h after intraperitoneal injection (a), the correlation between the concentration in hippocampus and blood concentration (b), the correlation between the concentration in the striatum and blood concentration (c), and the correlation between the concentration in cortex and blood concentration (d).

**Table 1:** Optimized mass spectrometry conditions of scopolamine with internal standard.

Compound	Precursor ion (*m*/*z*)	Product ion (*m*/*z*)	Declustering potential (V)	Collision energy (V)
Scopolamine	304.2	138.1	53	30
		156.1	53	30
		120.9	53	30

Pseudoephedrine (IS)	166.3	148.1	44	15

**Table 2:** Calibration curves and lower limits of quantification.

Sample	Liner range (ng/mL)	Regression equation	*r*	LLOQ (ng/mL)
Plasma	2∼2500	*y* = 0.01194*x* + 0.01249	0.996	2
		*y* = 0.01016*x* + 0.03244	0.994	
		*y* = 0.01305*x* + 0.00202	0.992	

Brain homogenate	2∼2500	*y* = 0.01108*x* + 0.01998	0.996	2
		*y* = 0.01034*x* + 0.00890	0.993	
		*y* = 0.01095*x* + 0.00723	0.997	

**Table 3:** Accuracy and precision.

Sample	Nominal conc. (ng/mL)	Intraday batch		Interday batch	
		Accuracy (%, RE)	Precision (%, RSD)	Accuracy (%, RE)	Precision (%, RSD)
Plasma	2	111.36	4.75	118.89	1.03
	5	98.78	7.61	110.50	1.18
	250	112.16	12.94	112.46	12.38
	1875	103.25	14.12	107.27	11.06

Brain homogenate	2	109.92	4.84	87.72	3.98
	5	97.33	10.74	107.32	1.57
	250	114.35	14.60	109.96	4.04
	1875	93.23	2.58	94.10	10.65

**Table 4:** Matrix effect and recovery.

Sample	Nominal conc. (ng/mL)	Matrix effect (%)		Recovery (%)	
		(Mean ± SD), *n* = 6	RSD	(Mean ± SD), *n* = 6	RSD
Plasma	5	96.12 ± 5.56	5.79	185.99 ± 25.52	13.72
	1875	87.13 ± 3.65	4.09	142.81 ± 14.08	9.86

Brain homogenate	5	114.01 ± 13.00	11.40	155.04 ± 20.73	13.37
	1875	99.81 ± 6.79	6.81	92.87 ± 5.65	6.08

**Table 5:** Refrigeration stability.

Sample	Nominal conc. (ng/mL)	Refrigerated for 24 h (4°C)		Refrigerated for 48 h (4°C)	
		Accuracy (%, RE)	Precision (%, RSD)	Accuracy (%, RE)	Precision (%, RSD)
Plasma	5	106.72	3.81	109.36	5.32
	1875	108.41	2.53	114.18	8.61

Brain homogenate	5	93.93	4.05	106.84	4.78
	1875	111.58	1.58	91.25	11.20

**Table 6:** Repeated freeze-thaw and autosampler stability.

Sample	Nominal conc. (ng/mL)	One freeze-thaw cycle		Two freeze-thaw cycles		Autosampler (12 h)	
		Accuracy (%, RE)	Precision (%, RSD)	Accuracy (%, RE)	Precision (%, RSD)	Accuracy (%, RE)	Precision (%, RSD)
Plasma	5	109.45	3.21	143.99	9.45	87.22	7.88
	1875	97.46	2.21	114.27	3.93	99.73	9.82

Brain homogenate	5	115.70	9.44	106.54	1.07	117.94	4.33
	1875	91.09	3.01	86.23	6.35	113.22	3.25

## Data Availability

The data generated and analyzed in this study are available from the corresponding author on request.
